# Internet of Medical Things (IoMT)-Based Smart Healthcare System: Trends and Progress

**DOI:** 10.1155/2022/7218113

**Published:** 2022-07-16

**Authors:** Jyoti Srivastava, Sidheswar Routray, Sultan Ahmad, Mohammad Maqbool Waris

**Affiliations:** ^1^Department of Computer Science and Engineering, School of Engineering, Indrashil University, Rajpur, Mehsana, Gujarat, India; ^2^Department of Computer Science, College of Computer Engineering and Sciences, Prince Sattam Bin Abdulaziz University, Alkharj 11942, Saudi Arabia; ^3^Department of Mechanical Engineering, Adama Science and Technology University, Adama, Ethiopia

## Abstract

Internet of Medical Thing (IoMT) is the most emerging era of the Internet of Thing (IoT), which is exponentially gaining researchers' attention with every passing day because of its wide applicability in Smart Healthcare systems (SHS). Because of the current pandemic situation, it is highly risky for an individual to visit the doctor for every small problem. Hence, using IoMT devices, we can easily monitor our day-to-day health records, and thereby initial precautions can be taken on our own. IoMT is playing a crucial role within the healthcare industry to increase the accuracy, reliability, and productivity of electronic devices. This research work provides an overview of IoMT with emphasis on various enabling techniques used in smart healthcare systems (SHS), such as radio frequency identification (RFID), artificial intelligence (AI), and blockchain. We are providing a comparative analysis of various IoMT architectures proposed by several researchers. Also, we have defined various health domains of IoMT, including the analysis of different sensors with their application environment, merits, and demerits. In addition, we have figured out key protocol design challenges, which are to be considered during the implementation of an IoMT network-based smart healthcare system. Considering these challenges, we prepared a comparative study for different data collection techniques that can be used to maintain the accuracy of collected data. In addition, this research work also provides a comprehensive study for maintaining the energy efficiency of an AI-based IoMT framework based on various parameters, such as the amount of energy consumed, packet delivery ratio, battery lifetime, quality of service, power drain, network throughput, delay, and transmission rate. Finally, we have provided different correlation equations for finding the accuracy and efficiency within the IoMT-based healthcare system using artificial intelligence. We have compared different data collection algorithms graphically based on their accuracy and error rate. Similarly, different energy efficiency algorithms are also graphically compared based on their energy consumption and packet loss percentage. We have analyzed our references used in this study, which are graphically represented based on their distribution of publication year and publication avenue.

## 1. Introduction

The Internet of Things (IoT) deals with various interconnected computing devices, machines, objects, humans, or animals with unique IDs and is capable of transferring data within the network without human intervention [1]. It includes monitoring and controlling systems that enable smart homes, for example, thermostats, heating, ventilation, and air conditioning devices, including IoT. IoT can also be used in other domains like transportation, healthcare, industrial automation, and energy response to natural and man-made disasters. Various IoT applications in different domains are illustrated in Figure 1. Verma et al. [2] proposed a data congestion monitoring system having a sharp area structure, where IoT helps in convincing the control of the leading body in traffic area via advanced systems. Fuqaha et al. [3] presented the use of IoT for checking environmental conditions with the help of disappointment figures, sullying control, and alarm trigger under crisis.

The applications of IoT in healthcare are the most demanding areas of research as per the current scenario. The Internet of Medical Thing (IoMT) is playing a crucial role within the healthcare industry to increase the precision, consistency, and throughput of the electronic devices as presented by Joyia et al. [4]. Because of the current pandemic situation, it is highly risky for an individual to visit the doctor for every small problem. Hence, using IoMT devices, we can easily monitor our day-to-day health records, and thereby initial precautions can be taken on our own.

An IoMT-based smart healthcare system is a collection of various smart medical devices connected within the network through the internet. An IoMT framework-based smart healthcare is formed of various phases. Firstly, medical data will be collected from the patient's body using smart sensors integrated within smart wearable or implanted devices that are connected together via a body sensor network (BSN) [5] or wireless sensor network (WSN) [6]. Then, this data will be transferred over the internet to the next component dealing with the prediction and analysis phase. After receiving the medical data, analysis can be done using a proper AI-based data transformation and interpretation technique [7]. In case of serious problems, doctors or other medical requirements can be approached with the help of smart AI-based applications in smartphones [8]. In nonserious cases, self-preventive measures can be taken.

AI provides the capability to a computer or robot, which is controlled by a computer system for performing tasks that are usually done by humans via their intelligence. Within a smart healthcare system with proper data interpretation techniques, a machine can also monitor health parameters using the implanted/wearable sensors on the body of the person under observation. Real-time disease management and prevention with improved user-end experience can be achieved using AI. SHS deals with very sensitive medical data of the person under observation. Hence, providing essential security measures in IoMT-based SHS is a very crucial task. AI can also be used for providing security in IoMT by detecting network intrusion [9] and intermediate security attacks within the IoMT systems [10], performing web-based security assessment using an IoMT-SAF device [11], etc. In an emergency situation, an automatic alert can be given to different parties using AI, which will help in saving a life by taking immediate actions [12]. Hence, doctors can easily manage patients' records and can also provide off-time medical services using AI. Blockchain can also be used for providing security in an IoMT network. It is a distributed database that maintains secure and decentralized information electronically in a digital format, which will guarantee the security and fidelity of data. Hence, it generates trust without the involvement of a third party. Blockchain can be used in IoMT for providing security in medical servers with electronic health records like MedRec that can be used for permission and access control management of medical data [13].

Various advancements in the smart home technology provide a healthy life and enhanced healthcare quality, especially for the handicapped and elderly personalities, and these advancements provide a comfortable lifestyle for patients in homecare, thus avoiding their admittance to hospitals, nursing facilities, or other confinement facilities [14, 15]. SHS will improve healthcare facilities for humans from various locations outside the hospital [16], thereby reducing depression, stress, and loneliness inside hospital wards. Doctors can also monitor and diagnose patients' health parameters and provide medicine prescriptions accordingly from any location [17]. Also, the exponential improvement of various new software and hardware technologies in SHS helps people, especially the disabled ones, to easily access certain home appliances using various smart devices, such as smartphones, laptops, tablets, etc. SHS is made of various computing devices that act proactively on behalf of persistent users [18]. Hence, for making good decisions in SHS, we require essential features, for example, users' preferences need to be considered for finding their choice of interest in certain scenarios [19–24]. Here, user preferences deal with the information used for describing the situation of a person considering the physical medical status or requirements. In modern SHS, we measure and record specific health parameters, such as blood pressure (BP), body temperature, pulse, glucose level, etc. We can also send a reminder in SHS to patients for medications based on some prior input provided by the user.

Therefore, we are motivated to do a comparative analysis of various research challenges faced by different researchers while developing an IoMT-based SHS. Considering the sensitivity of the real-time medical environment, we are encouraged to work in the direction of an artificial intelligence-based smart healthcare system using the IoMT framework.

The major contributions of the research work are as follows:

1. To analyze various IoMT architectures used in AI-based smart healthcare system
2. To present a comparative analysis of various data collection techniques to improve the accuracy of collected medical data
3. To present a comprehensive analysis of various energy-efficient techniques to optimize energy consumption by IoMT devices in SHS
4. To explore various health domains of the IoMT framework along with their application in the smart healthcare system, including the types of sensors used for each domain
5. To propose various research challenges that need to be considered while creating an IoMT-based smart healthcare system

The rest of the paper is organized as follows: Section 2 represents the distribution of referenced papers based on the publication year and avenue, graphically.  Section 3 discusses various existing IoMT architectures used by various authors for SHS, gives a comparative analysis of various data collection techniques used in smart healthcare systems, and provides a comparison of different energy-efficient algorithms using various parameters.  Section 4 defines the health domain with its application in SHS.  Section 5 describes the findings of literature survey in terms of the concerned challenges during the design of an IoMT network.  Section 6 is the conclusion of the research work done through this paper.

## 2. Statistical Distribution of Publications Referred

Figure 2 compares the referenced papers according to the publication venue. Figure 2 highlights the distribution of referenced papers based on the type of journal. 67 papers from the total referenced papers are primary research papers from reputed journals, whereas 31 papers originate from conferences.

Figure 3 represents the frequency of papers concerning the smart healthcare system. We have reviewed only 7 papers that are published on or before the year 2014 because of our interest in recent technologies in this era. We have referenced 4 papers from the year 2015, whereas the year 2016 contains 10 research papers on energy efficiency, security, and accuracy of healthcare data. We expect modern technology-based quality paper growth in the IoMT system from 2017, with the papers becoming freely available from various reputed journals for reference. As it can be seen, we have referred to most of the recent papers to get updated regarding the current tools and technologies in this era.

## 3. Related Work

This section gives the comparative and comprehensive analysis of work done by various authors in IoMT-based Smart Healthcare systems regarding different IoMT architectures, data collection techniques, their comparative analysis, and a comparison of various energy-efficient algorithms.

### 3.1. IoMT Architectures

An IoMT-based smart healthcare system is a collection of various smart medical devices connected within the network through the internet [25]. An IoMT framework-based smart healthcare is formed of various phases. Firstly, medical data will be collected from the patient's body using smart sensors integrated within the smart wearable or implanted devices that are connected together via BSN or WSN [26]. Then, this data will be transferred over the internet to the next component dealing with the prediction and analysis phase. After receiving the medical data, analysis can be done using a proper AI-based data transformation and interpretation technique [27]. In case of serious problems, doctors or other medical requirements can be approached with the help of smart AI-based applications in smartphones [28]. In nonserious cases, self-preventive measures can be taken.

Sun et al. [29] explained that IoMT architecture mainly consists of 3 layers, which are as follows: the application layer, perceptual layer, and network layer. They are demonstrated in Figure 4. The bottom layer, i.e., the perceptual layer, deals with the collection of data from the source and making important viewpoints from the collected data. Now, the perception layer consists of 2 sublayers, i.e., the data access sublayer and data acquisition sublayer. Perception from the collected data is the main task done by the data acquisition sublayer, for which it utilizes various medical perception equipment and signals acquisition equipment. Graphic code, RFID, GPRS, etc., can be considered the major signal acquisition methods. The data access sublayer connects the collected data from the data acquisition layer to the network layer through short-range data transfer techniques, such as Bluetooth, Wireless Fidelity (Wi-Fi), ZigBee, etc.

The middle layer, i.e., the network layer, deals with providing various platform and interface-related services and provides various data transmission techniques. This layer is formed of 2 subsequent layers, namely, the service layer and the network transmission layer. The network transmission sublayer uses mobile communication networks, wireless sensor networks, internet, etc., for transmitting the data received from the perception layer in a precise, consistent, real-time, and barrier-free way. However, the service layer realizes the integration of various networks, information description formats, data warehouses, etc. For such integrations, it provides open interface services and various other platform-related services.

The application layer utilizes the information gathered from the network layer to manage the medical record by means of various applications. This layer again consists of 2 sublayers, namely, the medical information decision-making application layer and the medical information application layer. The medical information application layer contains various health care equipment and other materials related to information for maintaining patient information, such as inpatient, outpatient, medical treatment, etc., records, whereas the medical information decision-making application layer deals with the analysis of various pieces of information, such as patients, disease, medication, diagnosis, treatment, etc.

Sun et al. [1] explained another three-tier architecture with medical server level, sensor level, and personal server level. Sensor level contains various sensors and medical devices in the form of a local network like a body sensor network (BSN) using low power wireless technology (such as BLE, NFC, or RFID) to transfer data.

The personal server level has few personal servers that can internally process and store from smart wearable devices (like a smartwatch) or off-body devices (like routers). It is required in situations where either a network connection is lost or the user needs the patient's data remotely. The last layer is the medical server layer, which consists of an algorithm or program for early diagnosis, rehabilitation progress assessment, or continuous patient monitoring (for example, MobiCare and BSN-Care [30]). The problem stated here is security negligence.

Kumar et al. [31] proposed an end-to-end architecture named mHealth System that connects the IoT smart sensors directly with SHS. This architecture contains three layers, i.e., the data processing layer, data collection layer, and data storage layer. The bottom layer, i.e., the data collection layer, consists of IoT devices that can sense and collect medical parameters. The next layer, i.e., the data storage layer, stores medical data on wide-scale and high-speed storage racks. The topmost layer, i.e., the data processing layer, involves various techniques to analyze collected sensor data.

Abdulmohsin Hammood et al. [32] proposed the four-tier architecture of an Internet of Medical Thing health-based model, where the first tier is the WBSN tier in which sensors like ECG (Electrocardiography) are directly connected to the human body. Fetched data from these sensors are transferred to the coordinator node via wireless 802.15.6 standard, which is then transmitted to the next tier. Tier 2 is the Smart\Wireless technology interface tier, where smart devices are utilized for data inspection and analysis and then transfer this data to tier 3 either by smart devices or wireless communication technologies. Tier 3 is the infrastructure internet tier that provides various communication technologies. Tier 4 is the care-services tier, where the received data are forwarded to the intelligent server (IS), where the data are stored, analyzed, and forwarded for smart medical services.

Here, we have seen 4 architectures for an IoMT-based smart healthcare system, where most of them have three layers. The last architecture alone, proposed by Abdulmohsin Hammood et al. [32], has a four-tier architecture. Upon comparing all these architectures, we can generalize that the bottom-most layer will have sensors in direct contact with the human body. In the middle of the architecture, we need a few layers for the inception, storage, and processing of data. The topmost layer will be used for providing services to the end-users.

### 3.2. Technologies Used for the Collection of Sensor-Based Medical Data

IoMT-based SHS uses various techniques to collect and transfer sensor data to servers, such as BSN, WSN, or RFID [33]. BSN is an IOT-based technology in a healthcare system that deals with monitoring the health of patients using a collection of various wireless sensor nodes with low-weight and low-power consumption [34, 35]. BSN-based social insurance systems can be used for therapeutic administration systems to accomplish various security essentials [36]. Since BSN nodes collect sensitive information and may operate in a heterogeneous environment, they require strict security mechanisms like BSN-Care [30].

RFID is a contactless technique for the automatic identification of targets using radiofrequency with 2-way data communication in various zones identified by their unique names [37, 38]. RFID consists of 3 parts, namely, the reader, database management system, and radio frequency electronic tag [39]. It can be used for identifying locations, the management of medical equipment and assets, waste tracking, personal identification, and for the collection of vital sign data of patients, such as ECG and blood pressure data [40, 41]. The advantage of using RFID is that without any human intervention, it can recognize objects at long distances with strong anti-interference. Flexible RFID tags can be used to expand their reading range [31]. A low-cost inkjet-printed RFID tag antenna can be used in remote healthcare applications [42]. We can also work upon the middleware providing an interface between the reader-writer and backend application. It will capture data from the sensing device and conduct proofreading, filtering, processing, and transferring them to RFID [43]. It will make healthcare more affordable and convenient to use.

Wireless sensor network (WSN) is a network of different monitoring sensors located in a homogeneous or heterogeneous environment. WSN can be used in IoMT for monitoring the real-time physiological condition of the person under observation [44]. Also, there are sensors that can measure the pressure level by examining the body's perspiration, speed of movement, and temperature of the patient's body [45]. Dhunna et al. [46] proposed a smart grid monitoring application for providing security in WSN with very low energy consumption. Yadav et al. [47] proposed a clustering algorithm for minimizing the energy consumption within the WSN network.

### 3.3. Comparison of Data Collection Techniques

A smart healthcare system will work precisely only when it will get correct and accurate data [48]. Hence, this section elaborates on a comparative analysis of different smart healthcare data collection techniques to maintain the accuracy of collected medical data [49]. In Table 1, we have compared different research works done on the techniques that can be used for collecting sensitive medical data using parameters, such as accuracy, error rate, and correlation prediction. Tekieh et al. [50] used a survey to demonstrate the uses of data mining in the healthcare system. The main problem is to maintain the quality and security of a large amount of health-related medical data, which is progressively increasing every day [55]. To overcome the problem, they have discussed 3 data mining processes in brief, i.e., association, clustering, and classification. They have discussed 4 applications of these techniques of data mining in SHS, i.e., the health of a population, health administration and policies, biomedicines and genetics, and clinical decision-taking [56].

Shahin et al. [51] proposed an advanced reduction technique named dynamic rough sets attribute reduction (DRSAR) with multiple classifiers for a random forest (RF) in the healthcare information systems (HIS). This model will be helpful to overcome the most critical challenges, i.e., for extracting relevant information from a large amount of medical data that needs to support the proper working of the system. The efficiency of the model is examined using 4 case studies (namely, premature birth, coronary heart disease, osteoporosis, and acute appendicitis). They have also provided web interfaces so that patients can calculate the level of risk involved with every medical case.

Yang et al. [52] proposed an association rule remining algorithm, multimode, and high-value association rule mining (MH-ARM) based on both the characteristics of data and the user's intention and knowledge as shown in Figure 5. They have considered more metrics, such as Kulczynski (KULC) and imbalanced ratio (IR), for the measurement of the support-confidence framework. They have taken 2 threshold values, i.e., the minimum support and minimum confidence, and they can be adapted as per the need of the user.

#### 3.3.1. Multimode Association Rule Mining

Let A and B be the attributes that can be shared for every instance belonging to the same class or unshared specific attribute varying with every instance. Then, multimode association rule mining can be given by Figure 6.

Here, four parameters are used, namely, support, confidence, correlation, and novelty, to extend the support-confidence framework of association rules given in equation (1). KULC and IR will provide the support and confidence for the algorithm, whereas novelty is calculated in equation (4), and the overall weight for the association rule remining algorithm, multimode, and highvalue association rule mining (MH-ARM) is calculated in equation (5).

(1) $$\begin{array}{c} X\Rightarrow Y\left[\sup,\text{conf},\text{corr},\text{novelty}\right], \end{array}$$

where sup represents the support of the algorithm and is calculated with the help of IR. Similarly, conf represent the confidence of the algorithm and is calculated with the help of KULC.

KULC: given 2 item sets *X* and *Y*, and KULC of *X* and *Y* can be calculated as follows:

(2) $$\begin{array}{c} KULC\left(X,Y\right)=\frac{1}{2}\left(P\left(X|Y\right)+P\left(Y|X\right)\right). \end{array}$$

From (2), we can say that KULC is subjective to the conditional probability of *P*(*X|Y*) and *P*(*Y|X*) and is independent of the number of records. The value of KULC will be from 0 to 1. The higher value of KULC signifies greater relevance between *X* and *Y*.

IR: the imbalanced ratio for *X* and *Y* can be calculated using

(3) $$\begin{array}{c} IR\left(X,Y\right)=\frac{\left|\sup\left(X\right)-\sup\left(Y\right)\right|}{\sup\left(X\right)+\sup\left(Y\right)-\sup\left(XUY\right)}. \end{array}$$

If both *X* and *Y* are in the same direction, then *IR*(*X*, *Y*) is 0. Otherwise, the increase in the difference of two directions gives a higher *IR* value. As it can be seen from equation (3), *IR* is independent of zero transaction and number of records.

Novelty: novelty rules neither inferred by others nor known to the users. Rule *x*⇒*y* will be treated as novel when *P*(*XY*) cannot be inferred by *P*(*X*) or *P*(*Y*). Novelty can be refined using

(4) $$\begin{array}{c} \text{Nov}\left(x\Rightarrow y\right)=\frac{P\left(XY\right)-P\left(X\right)P\left(Y\right)}{P\left(X\right)P\left(Y\right)}. \end{array}$$

For the determination of weights, they have used analytic hierarchy process (AHP) using “support—confidence—correlation—novelty” as a comparison parameter, with the weights of C, S, K, and N being 0.482, 0.11, 0.19, and 0.218, respectively. Therefore, the complete evaluation coefficient obtained is given in

(5) $$\begin{array}{c} R=0.482*C+0.11*S+0.19*K+0.218*N. \end{array}$$

Electronic health record system helps in the storage and organization of data. Mdaghri et al. [53] used this technique with data mining approaches to gain accuracy during the extraction of information from huge raw data. They elaborate on the application of data mining in healthcare, especially for the following four categories: the health of a population, health administration and policies, biomedicines and genetics, and clinical decision making. Roy et al. [54] proposed a variation of the decision tree model using the correlation ratio (CR) concept for smart healthcare datasets with many attributes, and each attribute contains various values. They have applied this model to various healthcare datasets to prove that the correlation ratio-based approach is unbiased toward a number of attributes, thereby giving more accuracy to the result.

Suppose *l* tuples are available in a dataset and the number of times *y* ∈ *Y* (where *Y* is set of outcomes) occurs is *l*_*y*_, then the dataset partitioned by their outcomes is given by

(6) $$\begin{array}{c} \forall y\in Y|\left\{S_{y}=\left(x_{jy}^{\left(1\right)},\ldots ,x_{jy}^{\left(n\right)}\right)\right\};j=1,\ldots ,l_{y}, \end{array}$$

where *S*_*y*_ is the set of tuples with the outcome *y*, and *j* is the value for the *i* − *th* attribute of the *j* − *th* tuple among all the *l*_*y*_ tuples with the outcome *y*. Equation (7) shows the average of the *i* − *th* attribute from all the tuples in each outcome class.

(7) $$\begin{array}{c} \forall y\in Y|\bar{x_{y}^{\left(i\right)}}=\frac{\sum_{j=1}^{l_{y}}x_{jy}^{\left(i\right)}}{l_{y}}. \end{array}$$

Equation (8) gives the overall average for the *i* − *th* attribute of all tuples.

(8) $$\begin{array}{c} \bar{x^{\left(i\right)}}=\frac{\sum_{y\in Y}\sum_{j=1}^{l_{y}}x_{jy}^{\left(i\right)}}{l}\\ =\frac{\sum_{y\in Y}l_{y}{\bar{x}}_{y}^{\left(i\right)}}{l}. \end{array}$$

The square of CR between the *i* − *th* attribute and outcome (class attribute) is given by

(9) $$\begin{array}{c} Cr_{\left(i\right)}^{2}=\frac{\sum_{y\in Y}l_{y}{\bar{x}}_{y}^{\left(i\right)}-\bar{x^{\left(i\right)}}2}{\sum_{y\in Y}\sum_{j=1}^{l_{y}}{\left({\bar{x}}_{jy}^{\left(i\right)}-{\bar{x}}^{\left(i\right)}\right)}^{2}}. \end{array}$$

Now, this CR will be able to find nonlinear dependencies, which will reflect the biasness, and thereby improve the accuracy of the collected data, whereas in paper [34], a detailed analysis of the physician and hospital rating data was done using a toolkit based on open-source modules, which are the publicly available datasets of USA.

### 3.4. Comparison of Energy Efficiency Measurement Techniques

Energy efficiency determines the size, lifetime, and usability of IoMT-based medical devices used in SHS [57, 58]. Implant devices should have a battery life minimum of 10 years to 15 years to avoid repetitive surgery as it results in physical and financial loss [59]. As far as wearable devices are considered, frequent battery changes reduce device usability [60]. Energy efficiency can be measured through various parameters, such as the amount of energy consumed, packet drop ratio, delivery time, data leakage, energy discharge, battery lifetime, packet loss, QoS (Quality of Service), power drain, network throughput, end-to-end delay, transmission rate, outage probability, internode distance, path-loss, and antenna gain. As shown in Table 2, Rehman et. al. [7] have compared their energy-efficient IoT e-health model with the attribute-based encryption (ABE) and privacy-enhanced data fusion system (PDFS) model using parameters EC (energy consumption), PDR (packet drop ratio), DT (delivery time), and DL (data leakage). For reducing latency by minimizing the number of hops, they use the heuristic formula, *h*(*n*)=*d*+*t*_*d*_, for each node, where *t*_*d*_ is the delivery time and distance *d* is comprised of distance from source node *i* to corresponding neighbor *n*_*i*_, which is denoted by *d*′. *d*_edge is the distance of the neighbor to the corresponding network edges *edge*_*i*_, and thereby, the mobility ratio for the network edge is given in

(10) $$\begin{array}{c} {\text{edge}}_{m},d=\frac{1}{\left(d^{\prime }+d_{\text{edge}}+{\text{edge}}_{m}\right)}. \end{array}$$

Now, the calculation of *t*_*d*_ includes delay time and data reception fluctuations, denoted by *d*_recp_. This model sets a threshold value to determine the strong *s* and weak *ω* transmission channel *c*, which is given as follows:

(11) $$\begin{array}{c} \left\{\begin{array}{c} \text{if}d_{\text{recp}}>\text{threshold,}\\ \text{then}c=s,\text{else}c=\omega . \end{array}\right. \end{array}$$

They proved through simulation results that the proposed model, when compared with ABE and PDFS, respectively, has improved the efficacy by 13% and 15% for data latency, 19% and 21% for packet drop ratio, 16% and 18% for energy consumption preround, 21% and 28% for delivery time, and 12% and 14% for data breaches.

Sodhro et al. [63] proposed an energy-efficient algorithm (EEA) that mainly focuses on data transmission and connectivity increase with a reduced interruption during information transfer. The authors compared the proposed algorithm with battery recovery-based lifetime enhancement (BRLE) using parameters, such as energy dissipation and charge dissipation. The discharge curve for the battery is defined by the voltage function, which includes the state of charge (SOC) with exponential decay. (12) and (13) show the discharge curve by SOC, which is equal to *st*, and *S* gives the remaining capacity/total capacity.

(12) $$\begin{array}{c} F\left(V\right)=st*\frac{e^{-\beta^{2}\left(t_{k}-t_{f}\right)}-e^{-\beta^{2}\left(t_{k}-t_{i}\right)}}{\beta^{2}}, \end{array}$$

(13) $$\begin{array}{c} F\left(V\right)=S*\frac{e^{-\beta^{2}\left(t_{k}-t_{f}\right)}-e^{-\beta^{2}\left(t_{k}-t_{i}\right)}}{\beta^{2}}, \end{array}$$

where *F*(*V*) denotes the voltage function of battery, *S* is the state of charge, *t* denotes the time duration for battery discharge, *β* is the parameter used for battery diffusion, *t*_*k*_ is the time duration of task *k*, *t*_*f*_ is the time for turning ON the load, and *t*_*i*_ is the time for turning OFF the load. They have shown through MATLAB simulation that EEA dissipates 89.7 J of energy, while BRLE dissipates more energy up to 95.68 J, and the charge dissipation of EEA is only 16,657.1409 mC·mint, while that of BRLE is 18,742.6591 mC·mint.

Lazarevska et al. [65] proposed a routing protocol for low power and lossy networks (RPL) to provide energy efficiency while accounting for the mobility of sensor nodes in WSNs with both static and mobile nodes. The proposed model objective function considers 5 parameters: EC (energy consumption), PDR (packet delivery ratio), duty cycle, total control overhead, and network lifetime. For calculating network lifetime, they used the power tracker tool for online monitoring of real-time duty cycle providing average simulated radio duty cycles of the transmission (Tx) and reception (Rx) of data for each node in (%) using

(14) $$\begin{array}{c} \text{Time}\_Rx=\frac{Rx\%}{100}.\text{Simulatio}n\_\text{Time,} \end{array}$$

(15) $$\begin{array}{c} \text{Time}\_Tx=\frac{Tx\%}{100}.\text{Simulation}\_\text{Time}. \end{array}$$

Using (16), the energy consumption of every single node and of whole network can be estimated.

(16) $$\begin{array}{c} E=P.t\\ =V.I.T, \end{array}$$

where *E* is energy, *P* is power, *V* is voltage, *I* is current, and *t* is the total time spent in a state. From equations (14), (15), and (16), we can reach

(17) $$\begin{array}{c} E\_rx=P\_rx\cdot \text{Time}\_rx=V\cdot I\_rx\cdot \text{Time}\_rx,\\ E\_tx=P\_tx\cdot \text{Time}\_tx=V\cdot I\_tx\cdot \text{Time}\_tx,\\ E\_\text{total}=E\_tx+E\_rx+E\_\text{cpu}+E\_\text{lpm}. \end{array}$$

Here, the predefined values for voltage, transmission, and reception current are 3 Volts, 8.5 mA, and 19.7 mA, respectively. The total energy consumption is given by the sum of the independent energy consumption of *Tx*, *Rx*, CPU (central processing unit) and *LPM* (low power CPU model). Now, *E*_cpu and *E*_lpm are relatively very small, and hence, they can be neglected easily for the final formula of the total average energy consumption as

(18) $$\begin{array}{c} E\_\text{total}=E\_tx+E\_rx, \end{array}$$

Tanzila et al. [66] proposed a secure and energy-efficient e-healthcare (SEF-IoMT) framework using the Internet of Medical Things (IoMT) and compared it with a simplified energy-balanced alternative-aware routing algorithm (SEAR), energy-efficient routing protocol (EERP), and critical routing data (CRD) using network simulator NS3. For measuring energy efficiency, they used five parameters, namely, packet loss rate, network throughput, energy consumption (EC), E2E (end-to-end) delay, and link breakages. The formula for calculating energy consumption is given in

(19) $$\begin{array}{c} E_{tx}\left(k,d\right)=E_{\text{elect}}*k+k*E_{fs}*d^{2},\\ E_{tx}\left(k\right)=E_{\text{elect}}*k, \end{array}$$

where *E*_*tx*_ shows transmitting energy, *E*_elect_ gives energy consumption per data bit, *E*_*fs*_ is energy for transmitted amplifier, *k* denotes data bits, and *d* shows the distance between the sensor nodes. In this algorithm, biosensors are interconnected through a undirected graph by the cost function *f*(*c*), which includes the weighted residual energy (*WRE*), number of sink hops *h*_*c*_, distance to neighborhoods *N*_*i*_, and queuing delay *Q*_*d*_ factors. The network throughput can be measured using

(20) $$\begin{array}{c} f\left(c\right)=w1*WRE+w2*\left(\frac{1}{h_{c}}\right)+w3*\left(\frac{1}{N_{i}}\right)+w4*\left(\frac{1}{Q_{d}}\right), \end{array}$$

where *w*1, *w*2, *w*3, *w*4 are weighted coefficients, and their summation is 1. Link breakage and packet loss can be calculated using

(21) $$\begin{array}{c} WRE=C_{e1}+C_{e2}+\cdots +C_{en}, \end{array}$$

(22) $$\begin{array}{c} C_{e}=\frac{\left(e_{\text{init}}-e_{tx}\left(k\right)\right)}{e_{\text{net}}}, \end{array}$$

where *C*_*e*1_, *C*_*e*2_,…, *C*_*en*_ is the estimated energy consumed with neighboring nodes, *e*_init_ is the initial energy, *e*_net_ shows network energy, and *e*_*tx*_(*k*) denotes the energy required for transmitting *k* data bits over a periodic time interval Δ*t*. The delay can be calculate using

(23) $$\begin{array}{c} Q_{d}=\frac{\left(a_{r}+t_{c}\right)}{D_{i}}, \end{array}$$

where *Q*_*d*_ is the queuing delay, *a*_*r*_ denotes arrival data packets *D*_*i*_ to sensor node *i*, and *t*_*c*_ shows the transmission capacity of the link.

Abdulmohsin Hammood et al. [32] proposed inter-WBAN cooperation in the IoMT environment (IWC-IoMT) for providing communication between wireless body sensor networks (WBSN) and those that are beyond their communication range. Efficiency comparison between the proposed algorithm and noninter-WBAN cooperation, namely, two hops in IoMT environment (TH -IoMT) and direct transmission in IoMT environment (DT-IoMT), is done. The formula for calculating the efficiency of DT-IoMT is as shown in

(24) $$\begin{array}{c} E_{i,j}=\left(1-P_{i,j}^{\text{out}}\right)\frac{\beta_{i,j}}{P_{i,j}^{tot}}\left[\frac{\text{bit}}{\text{joule}}\right], \end{array}$$

where *β*_*i*,*j*_ is the rate of data transmission from node *i* to *j*, *P*_*i*,*j*_^*tot*^ is the total power consumption, and the calculating formula is given in

(25) $$\begin{array}{c} P_{i,j}^{tot}=P_{amp}+P_{tx}+P_{rx}, \end{array}$$

where *P*_amp_ shows power consumption by amplifier for transmission, and *P*_*tx*_ and *P*_*rx*_ show power consumption by an internal circuit for transmission and reception, respectively.

The formula for calculating the efficiency of DT-IoMT is as shown in

(26) $$\begin{array}{c} E_{TH}=\frac{\left(1-P_{s1,cn1}^{\text{out}}\right)\left(1-P_{cn1,T2}^{\text{out}}\right)\beta \text{TH}}{P_{TH}^{tot}}. \end{array}$$

Here, *β*_TH_ is the rate of data transmission in DT-IoMT, *P*_*TH*_^*tot*^ is the total power consumption, and the calculating formula is given in

(27) $$\begin{array}{c} P_{TH}^{tot}=2\left(P_{\text{amp}}+P_{tx}+P_{rx}\right). \end{array}$$

Finally, the energy efficiency for IWC-IoMT of the 1^st^ sensor in the network is given by

(28) $$\begin{array}{c} Es=\frac{\left(1-P_{s1,cn1}^{\text{out}}\right)\left(1-P_{S1,cn2}^{\text{out}}\right)\beta_{\text{FH}}}{P_{\text{amp}}+P_{tx}+2P_{rx}}-\frac{\left(1-P_{cn1,T2}^{\text{out}}\right)\left(1-P_{cn2,T2}^{\text{out}}\right)\beta_{\text{SH}}}{2P_{\text{amp}}+P_{tx}+P_{rx}}. \end{array}$$

Here, (1 − *P*_*s*1,*cn*1_^out^)(1 − *P*_*S*1,*cn*2_^out^) represents the probability of successful transmission from *s*1 to *cn*1, and from *s*1 to *cn*2, respectively, and (1 − *P*_*cn*1,*T*2_^out^)(1 − *P*_*cn*2,*T*2_^out^) represents the successful transmission probability from *cn*1 to *T*2, and from *cn*2 to *T*2, respectively.

The first term total power, *P*_amp_+*P*_*tx*_+2*P*_*rx*_, contains two nodes for receiving data and one single node for transmitting data, however, in the second term total power, 2*P*_amp_+*P*_*tx*_+*P*_*rx*_ contains two data transmission nodes and a single data reception node. Now, *β*_FH_ shows the rate of data transmission from sensors to coordinators (first phase), and *β*_SH_ shows the data transmission rate from coordinators to *T*2 (second hop).

### 3.5. Performance Comparison

Figure 7 shows the comparison of the percentage of accuracy achieved by 6 decision tree classification models, namely, J48, iterative dichotomiser 3 (ID3), random forest (RF), correlation ratio (CR), information gain (IG), and gain ratio (GR). Here, the accuracy of RF is 97.71%, ID3 is 71.8%, J48 is 88.95%, IG is 70.83%, GR is 72.26%, and CR is 71.09%. It is clear from the graph that the multiclassifier random forest is giving the highest accuracy among all six algorithms.

Figure 8 shows the comparison of error rates for 3 machine learning decision tree classification algorithms, namely, J48, iterative dichotomiser 3 (ID3), and random forest (RF). Here, the error rate for ID3 is 28.19%, J48 is 11.04%, and RF is 2.28%. The graph clearly shows that the multiclassifier random forest gives a minimum error rate in comparison to other two algorithms.

Figure 9 shows a comparison of improvement in the percentage of energy consumed by 3 methodologies (secure and energy-efficient framework using Internet of Medical Things (IoMT) for e-healthcare (SEF-IoMT), routing protocol for low power and lossy networks (RPL) with a new objective function (NEWOF), and an energy efficient IoT e-health model using AI with homomorphic secret sharing). As the graph shows, we have maximum improvement in SEF-IoMT, i.e., 29%, followed by the energy efficient IoT e-health model using AI with homomorphic secret sharing with 17% of improvement in energy consumption, and the last one is the routing protocol for low power and lossy networks (RPL) with a new objective function (NEWOF), which gives 1.45% of energy consumption improvement.

Figure 10 shows the comparison of the improvement in the percentage of packet loss during transmission by 2 methodologies, namely, SEF-IoMT and energy efficient IoT e-health model using AI, with homomorphic secret sharing. As the graph shows, we have a maximum improvement in SEF-IoMT, i.e., 42%, followed by the second methodology, with a 17% improvement in packet loss during transmission within the network.

## 4. Health Domain and Its Application

As shown in Figures 11 and 12, there are mainly three modules that need to be monitored in a smart healthcare system, namely, homecare [15], selfcare, and acute care [31]. In a selfcare system, a person can monitor and access his own fitness through different wearable devices and take necessary actions to prevent diseases in the future [8, 71]. In the homecare system, the healthcare providers measure patients' health remotely, and if any problem arises, an alarm will be triggered to alert the doctor and the patient, and both of them collaboratively decide the action that needs to be performed [27, 72]. Acute care deals with critical situations, where urgent responses are required. It is usually used for elderly care wearable/implanted devices [30, 73].

Each domain uses different types of sensors or a combination of one or more sensors.  Table 3 shows various sensors that can be used in a smart healthcare system to detect vital parameters of the client. The first sensor is the accelerometer, which belongs to the selfcare domain. It is used to measure the change in the linear velocity, and it is helpful to detect the blood glucose level of the patient or the person under observation [8]and the change in the position of the patient [70] or any other body part of the patient [74]. A gyroscope detects the angular velocity, which will help in detecting human tilt, and it uses an alarm for the professionals to gain their attention whenever required [75]. The magnetometer detects the magnetic field and relative orientation. It is mostly used in elderly care devices in conjunction with gyroscopes and accelerometers [30]. The LM35 sensor changes its voltage according to the change in temperature and generally measures the body temperature of the individual under observation [30, 77], whereas DHT11 is used to measure the environmental temperature and humidity [76, 78]. LM35 consumes more energy compared to DHT11. A small chip named AD8232 analyzes the pumping stroke of heart muscles, which results in ECG (Electrocardiogram) [80, 82]. ECG analyzes heart signals, irrespective of the body state of the person under examination [71, 79], whereas MAX 30105 is an integrated optical sensor with 2 LEDs in a single photodetector, processing low noise analog signals in combination with Ardunio to monitor the heart rate between 1.8 V and 3.3 V [71, 79, 81]. ADXL335 is a body position sensor used to check the proper shoulder position to prevent various complications, such as pain, swelling, respiratory problems, etc.

As we have discussed in this section, various types of sensors can be used in the IoMT network based on the requirement of the system. Besides the selection of accurate application-specific sensor, there are various other aspects that are to be considered while developing an IoMT network, which we are going to discuss in Section 5.

## 5. Challenges within a Smart Healthcare System to be Considered during IoMT Network Design

AI provides the capability of a computer or robot, which is controlled by a computer system for performing tasks that are usually done by humans via their intelligence [28, 83]. In a smart healthcare system with proper data interpretation techniques, a machine can also monitor health parameters using the implanted/wearable sensors on the body of the person under observation [84, 85]. Real-time disease management and prevention with improved user-end experience can be achieved using AI [86, 87]. Designing an IoMT-based smart network is very complex because of the below-mentioned challenges that influence the designing techniques at every edge [88]. The routing protocol will govern the exchange of data between routers and gives information, enabling route selection between nodes [89, 90]. In a smart healthcare system, we collect very sensitive patient data using small and ultralow power IoMT devices [91, 92]. Hence, the mentioned challenges cannot be tackled within the implanted/wearable IoMT devices, however, they can be balanced in the network and protocol designing techniques with the consideration of effective network topology, power conservation, and channel effectiveness. Hence, the few points that are to be considered especially in IoMT network designs are as follows:

1. Body movements: the real challenge arises when there are changes in network topology because of the movement of the user under observation with on-body sensors or medical devices [93]. Hence, the routing protocol in IoMT must be adaptable to deal with such unpredictable challenges without compromising the quality of communication strength.
2. Temperature change: the main cause of the rise in the temperature of the IoMT devise is the absorption of radiations by the antennas and the power consumed by node circuitry [94]. This rise in the temperature of the wearable or implant devices can result in damage to tissues or other body organs of the user under observation. Hence, the considerations of (transmission and computation) the power consumption of IoMT devices are essential.
3. Energy efficiency: energy efficiency determines device size, lifetime, and usability. Hence, the routing protocol should optimize the energy consumption by the IoMT device. Implant devices should have a battery life minimum of 10 to 15 years to avoid repetitive surgery as it results in physical and financial loss [59]. As far as wearable devices are concerned, frequent battery changes reduce device usability.
4. Range of transmission: when the range of data transmission is short, having postural body movements leads to disconnection and repartitioning among sensor nodes in the IoMT system [5].
5. Heterogeneous environment: the routing protocol for SHS must be capable of handling challenges because of the heterogeneous environment of BSN applications (for example DexterNet) [83, 95].
6. QoS: when we deal with real-time BSN applications, such as ECG, it is very sensitive for data loss, and it is time critical [96]. Hence, accordingly, the quality of service requirements should be made to deal with such situations. Now, implanted smart sensors have fixed memory and computational capabilities. Hence, the routing protocol should adopt QoS measures [35].
7. Security: users' data is stored in the cloud for more accurate and faster responses to the patients being monitored using IoMT devices, however, this advancement can lead to the risk of user data being stored or abused [1, 97, 98].

## 6. Conclusion and Future Scope

This research paper gives an overview of the Internet of Medical things (IoMT) with an emphasis on various enabling techniques used in smart healthcare systems (SHS). Here, we have discussed various methodologies used in smart healthcare systems, such as radio frequency identification (rfid), artificial intelligence (ai), blockchain, etc. This paper provides a detailed description and comparison of various IoMT architectures being used by multiple authors for AI-based smart healthcare systems. A smart healthcare system will work precisely only when it will get correct and accurate data. Hence, we are presenting a comparative analysis of different smart healthcare data collection techniques to maintain the accuracy of collected medical data. For collecting these medical data, we are using implant/wearable IoMT devices on the body of the patient. Implant devices should have a battery life minimum of 10 years to 15 years to avoid repetitive surgery as it results in physical and financial loss. As far as wearable devices are concerned, frequent battery changes reduce device usability. Energy efficiency determines the size, lifetime, and usability of the IoMT devices. Hence, we are focusing on techniques used for energy optimization by the IoMT device. This paper provides a detailed comparison through both tabular and graphical methods showing the recent work done by various authors to maintain the energy efficiency of an IoMT network. For calculating the efficiency of a system, different parameters are being used, such as the amount of energy consumed, packet delivery ratio, battery lifetime, quality of service, power drain, network throughput, delay, transmission rate, etc. In this paper, we are providing different correlation-based equations for finding accuracy and efficiency within the IoMT-based healthcare system. We are also discussing various health domains of the IoMT framework, including the list of sensors with their application in measuring the health of the person under evaluation.

In this paper, we have presented seven key protocol design challenges that need to be considered during the implementation of an IoMT network-based smart healthcare system, namely, the regular body movement of the patient, change in the temperature of the health monitoring device, energy efficiency of the network, transmission range of the device, performance of the IoMT device in a heterogeneous environment, quality of service, and security. In this work, we have compared and elaborated work for the efficient use of energy, which is only one of the key challenges, and the other six challenges need to be explored and analyzed in the future. Considering the sensitivity of medical data, a deep analysis and future enhancement must be done for providing security to the system.

## Figures and Tables

**Figure 1:** Overall view emphasizing the role of IoT in different domains.

**Figure 2:** Distribution by the type of papers.

**Figure 3:** Distribution of reference papers by the year of publication.

**Figure 4:** IoMT architecture overview.

**Figure 5:** MH-ARM framework.

**Figure 6:** Multimode association rule mining.

**Figure 7:** Comparison for accuracy.

**Figure 8:** Comparison of error rates.

**Figure 9:** Comparison graph for energy consumption.

**Figure 10:** Comparison for packet loss.

**Figure 11:** Acute care and selfcare example [31, 70].

**Figure 12:** Home care example [8, 31].

**Table 1:** Comparison of different data collection techniques.

Sl. no.	Authors and publication years	Parameters	Data collection technique	Advantages	Disadvantages
1	Tekieh et al. [50], 2015	Accuracy	Electronic health record	Different techniques with their merits are described. Hence, based on the requirement of research, an optimal approach can be considered	No suggestion about any new technique

2	Shahin et al. [51], 2014	Error rate, accuracy	Electronic health record	Case study provided in this research for practical application	Applicable for specific environment

3	Yang et al. [52], 2016	Accuracy	Rule-based approach	Data gathering speed is improved through the proposed mechanism	Further work can be done to improve accuracy.

4	Mdaghri et al. [53], 2016	Accuracy	Support system for clinical decision	Accurate data collection	Improper handling of missing values

5	Roy et al. [54], 2016	Correlation, accuracy	Correlation-based ratio analysis	Healthcare-related specific information is gathered because of correlation	Have not considered missing values.

6	Rao et al. [34], 2016	Prediction, accuracy	Open dataset	Better visualization because of GUI	Missing values not considered

**Table 2:** Comparison of recent energy efficiency measurement techniques.

Sr. no.	Authors and publication years	Parameters	Efficiency measurement technique	Advantages	Disadvantages	Efficiency improved
1	Rehman et al. [7] (2021)	Energy consumption (EC), packet drop ratio (PDR), delivery time (DT), and data leakage (DL)	Comparison of proposed model (energy-efficient IoT e-health model using AI with homomorphic secret sharing) [7] with (attribute-based encryption) ABE [61] and (privacy-enhanced data fusion system) PDFS [62] using simulation	1. The maintainability of the disease diagnosis system is increased. 2. Provides trust for communication in integration with medical cloud.	1. Under high network load, PDR increased 2. No fixed energy consumption for all IoT nodes. 3. Lack of intelligence that is required for avoiding packet collision during the increased speed of edge nodes.	EC = 17% PDR = 20% DT = 24.5% DL = 13%

2	Sodhro et al. [63] (2021)	Energy dissipation (ED), charge dissipation (CD), energy discharge and battery lifetime	Comparison of proposed model (energy-efficient algorithm) [63]with (battery recovery-based lifetime enhancement) BRLE [64] using MATLAB simulation	1. It consumes low energy 2. Increased battery lifetime.	Computational load is high	ED = 6.67% CD = 12.52%

3	Lazarevska et al. [65] (2018)	Energy consumption (EC), network lifetime (NL), packet delivery ratio (PDR), and total control traffic overhead (TCTO)	Comparison of proposed new objective function (NEWOF) and minimum rank with hysteresis objective function (MRHOF) using powertracker tool in CoojaContiki OS.	1. Improvement in the total energy consumption. 2. Improvement in TCTO 3. Less degradation in PDR. 4. Energy efficiency improved	During the implementation of mobility plug-in, this model shows approximately 20% loss.	PDR = 3% EC = 1.45% NL = 8% TCTO = 5.8%

4	Tanzila et al. [66] (2020)	Network throughput (NT), packet loss rate (PLR), end-to-end delay (E2E), energy consumption (EC), and link breakages (LB)	Comparison of proposed algorithm SEF-IoMT [66] against existing solutions EERP [67], CRD [68], and SEAR [69] using NS3	1. Decrease energy consumption thereby providing more efficiency 2. Data delivery toward medical experts is increased. 3. Highly secure with validation and integrity support 4. Lower network delay	1. Improvement required in SEF-IoMT for mobility-based medical scenarios. 2. This framework requires the improvement of energy consumption and network security when dealing with inter-WBAN data transformation	NT = 18% PLR = 44% E2E = 26% EC = 29% LB = 48%

5	Abdulmohsin Hammood et al. [32]	Energy efficiency (EE), power consumption (PC), transmission rate (TR), outage probability (OP)	Comparison of the proposed algorithm inter-WBAN cooperation in an IoMT environment (IWC-IoMT) with noninter-WBAN cooperation (direct transmission in an IoMT environment (DT-IoMT) and two hops in an IoMT environment (TH-IoMT))	1. Greater energy efficiency of IWC-IoMT than DT-IoMT and TH-IoMT. 2. The outage probability of IWC-IoMT is higher than that of DT-IoMT and TH-IoMT during symmetric transmission.	During asymmetric transmission, the outage probability of IWC-IoMT degraded compared to DT-IoMT and TH-IoMT	EE = 10% PC = 2% (PC increased with increase in TR) TR = 3% OP = 5% (with internode distance >2.5 m)

**Table 3:** List of sensors and their application in the smart healthcare system.

Sr. no.	Name of sensors	Description	Applications	Belonging domain
1	Accelerometers	Measures acceleration	Detects glucose level in blood [8], human motion [70], and body movement [74].	Home care

2	Gyroscope	Detects angular velocity	Detects human tilt and provides an alert system for a problematic scenario [75].	Acute care

3	Magnetometer	Detects magnetic field and relative orientation	When used in combination with a gyroscope and an accelerometer, it is capable of detecting human fall, and it is mostly used in elderly devices [30].	Acute care

4	LM35	Senses body temperature	This sensor varies voltage with changes in temperature in centigrade [76–78]. It is used for measuring body temperature.	Selfcare

5	DHT11	Humidity and temperature sensor	This sensor can be used to measure temperature between 0°C and 50°C and humidity between 20% and 90%. It is a low-power consuming sensor with 5% accuracy [71, 77, 78]. It is used for measuring environmental conditions.	Selfcare/home care

6	AD8232	Electrocardiogram sensor	It analyzes heart signals, irrespective of the body state of person under examination [71, 79, 80].	Home care/acute care

7	ADXL335	Body position sensor	This sensor helps in proper positioning to prevent various complications, such as body sore, swelling, pain, or respiratory problems [71].	Selfcare

8	MAX 30105	Sensor monitors heart rate	This integrated optical sensor with 2 LEDs in a single photo detector processes low noise analog signal in combination with Ardunio to monitor heart rate in between 1.8 V and 3.3 V [71, 79, 81].	Selfcare/home care

## Data Availability

The data used to support the findings of this study are available from the first author upon request (jyotisrivastava688@gmail.com).
